# Investigation of the Mechanism of hsa_circ_000 1429 Adsorbed miR-205 to Regulate KDM4A and Promote Breast Cancer Metastasis

**DOI:** 10.1155/2022/4657952

**Published:** 2022-06-21

**Authors:** Yuting Xu, Cheng Qian, Chunxiao Liu, Yingqiang Fu, Kaiyuan Zhu, Zhenbo Niu, Jiaxin Liu

**Affiliations:** Department of Breast Cancer Surgery, Harbin Medical University Cancer Hospital, Harbin 150081, China

## Abstract

This study investigates the mechanism of hsa_circ_0001429 adsorbing miR-205 and regulating the expression of KDM4A to promote breast cancer metastasis and its mechanism. Mammary epithelial cells MCF-10A and human breast cancer cell lines BT474, SKBr-3, ZR-75-30, and MCF7 are cultured, and the mRNA expressions of hsa_circ_000 1429, miR-205, and KDM4A are detected by qRT-PCR; hsa_circ_000 1429 binds to miR-205, and miR-205 targets KDM4A. RIP verifies that hsa_circ_000 1429 binds to AGO2; RNA pull down results prove that hsa_circ_000 1429 binds to miR-205; MTT detects cell proliferation; transwell assay detects cell migration and invasion ability; flow cytometry detects cell apoptosis rate. The expressions of KDM4A, migration, and invasion-related factors, N-cadherin and MMP-9 protein, are detected by blot. hsa_circ_000 1429 may upregulate the KDM4A gene by adsorbing miR-205. Therefore, it will promote the proliferation, migration, and invasion of breast cancer cells and inhibit their apoptosis.

## 1. Introduction

Breast cancer is one of the most common malignant tumors in women in my country, and its morbidity and mortality are on the rise [1–4]. In recent years, new breast cancer targeted drugs have emerged one after another, which has significantly improved the prognosis of patients with early breast cancer. However, the prognosis of patients with locally advanced or metastatic breast cancer is still poor [5, 6]. At present, the molecular mechanism of breast cancer invasion and metastasis is still unclear, and finding new biological targets is of great significance for improving the prognosis of breast cancer patients. Circular RNAs (circRNAs) are newly discovered endogenous noncoding RNAs, which are hundreds or even thousands of bases in length and have a covalently closed structure [7, 8]. A large number of studies have shown that circRNAs can regulate a variety of cancer-related biological processes, including cell proliferation, invasion, and metastasis [9–11]. CircRNA exists widely in mammals and its content is stable, and it is one of the hotspots in the field of oncology [12, 13]. After reviewing the literature, the study finds only one literature reporting this circRNA. Chen et al. believed that hsa_circ_000 1429 is downregulated in breast cancer tissues and cells and could inhibit the proliferation, migration, and invasion of breast cancer cells [14, 15]. However, there is no research report on the regulatory relationship of hsa_circ_0001429 in the occurrence of breast cancer and the downstream regulatory network. The study finds a binding site between hsa_circ_000 1429 and miR-205 by querying the Shengxin website. miR-205 has a regulatory role in the occurrence of colorectal cancer, breast cancer, glial cell carcinoma, and other malignant tumors, but miR-205 has an opposite expression trend in different cancers [16, 17]. The regulatory mechanism of miR-205 expression in breast cancer is still inconclusive [18]. In addition, the study screens the downstream target genes of miR-205 through the StarBase website and finds that there is a binding site between miR-205 and KDM4A. There is no research report on whether miR-205 and KDM4A have a targeted regulatory relationship [19]. Studies have reported that KDM4A can promote the chemosensitivity of ovarian cancer cells [20]. Some studies have reported that KDM4A may act as a new breast cancer inhibitor, which can inhibit the development of breast cancer by inducing apoptosis of breast cancer cells. In this study, we aimed to explore the regulatory relationship of hsa_circ_0001429 in breast cancer by culturing breast cancer cells and processing them accordingly.

A biological prediction website is used to analyze the binding sites of miR-205, and it is verified that miR-205 can bind hsa_circ_000 1429 and KDM4A. The artificially synthesized hsa_circ_0001429 and KDM4A 3'UTR gene fragments are constructed into pMIR-REPORT. The complementary sequence mutation site of the seed sequence is designed and constructed into the pMIR-REPORT reporter plasmid. The correctly sequenced luciferase reporter plasmids WT and MUT are cotransfected with miR-205 into SKBr-3 cells (Shanghai Beinuo Biotechnology Co., Ltd.). 48 h after transfection, the luciferase activity is detected using the dual-luciferase reporter assay system (model: Promega E1910, Promega, USA).

Later, SKBr-3 cells in each group are transfected and cultured for 48 hours. The cells in each group are collected and counted as follows: 5 × 10^3^ cells per well are seeded into 96-well plates and cultured in an incubator. At 24 h, 48 h, and 72 h, 20 *μ*L of 5 mg/mL MTT solution is added to each well, and the culture is terminated after incubation at 37°C for 2 h. The culture supernatant in the wells is aspirated and discarded, and 150 *μ*L of DMSO is added to each well. The absorbance value of each well is read at 570 nm (optical density, OD) value.

The remainder of this study is organized as follows.  Section 2 presents the experimental method.  Section 3 provides the experimental result, and Section 4 illustrates the experimental result discussion. Finally, the conclusions of this study are given in Section 5.

## 2. The Proposed Method

The breast cancer cells are collected and lysed, and the cell extract is incubated with the antibody for coprecipitation. 50 *μ*L of magnetic beads are ished and resuspended in 100 *μ*L of RIP Ish buffer, and 5 *μ*g of antibody AGO2 (lot number: ab32381, 1 : 50, Abcam, UK is added.) and IgG (1 : 100, batch number: ab109489, Abcam, UK) is incubated. Magnetic bead-antibody complexes are ished and resuspended in 900 *μ*L RIP Ish buffer; add 100 *μ*L of cell extract and incubate overnight at 4°C. The samples are digested with proteinase K to extract RNA, and the expression level of hsa_circ_000 1429 is detected by qRT-PCR.

WT biotinylated and MUT biotinylated miR-205 breast cancer cells are transfected, cell lysates (lot number: ab95401, Abcam, UK) are lysed, and the lysates are mixed with precoated RNase-free, and yeast tRNA M-280 streptavidin magnetic beads (batch number: 112–06D, Invitrogen, USA) are incubated at 4°C for 3 h, ished twice with cold lysis buffer, and ished with low-salt buffer and high-salt buffer, respectively. After ishing 3 times and 1 time, the bound RNA is purified by TRIzol, and the expression level of hsa_circ_000 1429 is detected by qRT-PCR.

Cells are collected and lysed with RIPA lysis buffer (lot number: AR0105-30, Wuhan Boster Company), and then, the protein concentration is determined with the BCA protein quantification kit (70-PQ0012, Multisciences, Hangzhou, China). Proteins are dissolved in 2× SDS, separated by 10% SDS-PAGE, transferred to PVDF membrane, blocked with 5% nonfat milk powder at room temperature for 1 h, and ished with PBS for 2 min; the PVDF membrane is mixed with diluted primary antibodies KDM4A (1 : 1000, batch number: ab105400, UK Abcam Company), N-cadherin (1 : 1000, batch number: ab76057, UK Abcam Company), MMP-9 (1 : 1000, batch number: ab38898, UK Abcam Company), GAPDH (1 : 2000, batch number: ab 9485, UK Abcam Company) overnight at 4°C, ished 3 times with TBST for 5 min each, and incubated with 1 : 100 diluted HRP-labeled secondary antibody goat anti-mouse IgG antibody (batch number ab205719; 1 : 2000; Abcam, UK) for 1 h. It takes an ECL fluorescence detection kit (batch number: BB-3501, Ameshame, UK) with equal amount of solution A and solution B, mixes them in a dark room, drops them on the membrane, and puts them into a gel imager for exposure imaging. Photographs are taken with a BioRad image analysis system (model: Gel Doc XR+, BioRad, USA). GAPDH is used as an internal reference, and quantity is used as an internal reference.

Total RNA is extracted using the TRIzol kit (lot number: 15596026, Invitrogen, USA), according to the PrimeScript RT reagent kit (lot number: RR047A, TaKaRa, Japan). It is reverse-transcribed from total RNA into cDNA according to the instructions, and the Fast SYBR Green PCR kit (lot number: BL705A, Biosharp Company) and ABI PRISM 7300 RT-PCR system (model: ABI7300, American ABI Company) were used for qRT-PCR detection. Each experiment is repeated 3 times. Primer designs are given in Table 1.

The SPSS version 21.0 (IBM Corporation, USA) is used for statistical analysis. Measurement data are expressed as mean ± standard error $\left(\bar{x}\pm s\bar{x}\right)$, and the unpaired *t*-test is used for comparison between two groups. One-way ANOVA is used to compare data among multiple groups. According to Tukey's post hoc test, *P* < 0.05 indicates that the difference is statistically significant.

## 3. The Experimental Results

### 3.1. High Expression of hsa_circ_000 1429 and KDM4A in Breast Cancer Cells

The protein expression of KDM4A is detected by Western blot. Compared with mammary epithelial cells MCF-10A, hsa_circ_000 1429, KDM4A mRNA, and protein expressions are all elevated in human breast cancer cell lines BT474, SKBr-3, ZR-75-30, MCF7, and miR-205. The expression of hsa_circ_000 1429 in SKBr-3 is the highest (*P* < 0.05). It is selected as the cell verified by subsequent cytological experiments.  Figure 1 shows the expression of hsa_circ_000 1429, KDM4A, and miR-205 in breast cancer cells.

### 3.2. hsa_circ_000 1429 Adsorbed miR-205 to Regulate KDM4A

Compared with the NC mimic group, the luciferase activity of hsa_circ_000 1429 wild type and KDM4A wild type in the miR-205 mimic group specifically bound to miR-205. Both are inhibited (*P* < 0.05), while the luciferase activity of hsa_circ_000 1429 mutant and KDM4A mutant has no significant change (*P* > 0.05), indicating that miR-205 could bind to hsa_circ_000 1429 and KDM4A, respectively. Compared with the MUT-miR-205 and bio-NC groups, the expression of hsa_circ_000 1429 bound by WT-miR-205 is significantly increased (*P* < 0.05), indicating that miR-205 can be directly combined with hsa_circ_000 1429. In SKBr-3 cells, anti-AGO2 antibody could precipitate hsa_circ_000 1429, indicating that hsa_circ_000 1429 could form a complex with AGO2, thereby competitively binding to miR-205. The above results indicated that hsa_circ_000 1429 may regulate the expression of KDM4A gene by adsorbing miR-205 in breast cancer, as shown in Figure 2.

### 3.3. Silencing hsa_circ_000 1429 or Overexpressing miR-205 Inhibits Breast Cancer Cell Proliferation

In breast cancer cells SKBr-3, hsa_circ_000 1429 is silenced or miR-205 is overexpressed or miR-205 is silenced or KDM4A gene is overexpressed in hsa_circ_000 1429-silenced cells. Therefore, the study finds that hsa_circ_000 1429 may be activated by adsorption of miR-205, which regulates the effect of KDM4A on the biological activity of breast cancer cells. The proliferation of cells in each group is detected by MTT. Compared with the shRNA NC group, the proliferation ability of SKBr-3 breast cancer cells in the shRNA-hsa_circ_000 1429 group decreased at 48 h and 72 h (*P* < 0.05). Compared with mimics NC, the proliferation ability of breast cancer cells SKBr-3 in the miR-205 mimics group is significantly inhibited at 48 h and 72 h (both *P* < 0.05). The proliferation ability of breast cancer cells in the SKBr-3 inhibitor group and the shRNA-hsa_circ_000 1429 + pcDNA-KDM4A group is significantly increased (both *P* < 0.05). These results indicate that silencing hsa_circ_000 1429 or overexpressing miR-205 inhibited breast cancer cell proliferation.  Figure 3 shows the MTT assay for cell proliferation.

### 3.4. Silencing hsa_circ_000 1429 or Overexpressing miR-205 Inhibits the Migration and Invasion Ability of Breast Cancer Cells

Transwell assay is used to detect the migration and invasion ability of cells in each group. Compared with the shRNA NC group, the migration and invasion numbers of SKBr-3 breast cancer cells in the shRNA-hsa_circ_000 1429 group decreased (*P* < 0.05). Compared with the shRNA-hsa_circ_000 1429 group, the migration and invasion numbers of breast cancer cells in the SKBr-3 inhibitor group and the shRNA-hsa_circ_000 1429 + pcDNA-KDM4A group significantly increased (*P* < 0.05). These results indicate that silencing hsa_circ_000 1429 or overexpressing miR-205 inhibited breast cancer cell migration and invasion. The transwell assay to detect cell migration and invasion ability is shown in Figure 4.

### 3.5. Silencing hsa_circ_000 1429 or Overexpressing miR-205 Promotes Breast Cancer Apoptosis

Flow cytometry is used to detect cell apoptosis in each group. Compared with the shRNA NC group, the apoptotic rate of SKBr-3 breast cancer cells in the shRNA-hsa_circ_000 1429 group increased (all *P* < 0.05). Compared with the shRNA-hsa_circ_000 1429 group, the apoptosis rate of SKBr-3 breast cancer cells in the inhibitor group and shRNA-hsa_circ_000 1429 + pcDNA-KDM4A group significantly decreased. These results suggest that silencing hsa_circ_000 1429 or overexpressing miR-205 promotes breast cancer cell apoptosis.  Figure 5 shows that flow cytometry is used to detect cell apoptosis in each group.

### 3.6. hsa_circ_000 1429 Adsorbed miR-205 to Regulate KDM4A Expression and Inhibit Breast Cancer Metastasis

The mRNA and protein expressions of hsa_circ_000 1429 and KDM4A in breast cancer cells of the hsa_circ_000 1429 group significantly decreased. The expression of miR-205 and the protein expressions of migration and invasion-related factors N-cadherin and MMP-9 significantly increased (all *P* < 0.05). Compared to miR-205, there is no significant change in the expression of hsa_circ_000 1429 in breast cancer cells in the mimics group (*P* > 0.05). The expression of miR-205 significantly increases, the mRNA and protein expressions of KDM4A significantly decrease, and the protein expressions of N-cadherin and MMP-9 significantly increase (all *P* < 0.05). Compared with the shRNA-hsa_circ_000 1429 group, the expression of hsa_circ_000 1429 in the breast cancer cells of the shRNA-hsa_circ_000 1429 + miR-205 inhibitors group has no significant change (*P* > 0.05). The expression of miR-205 is significantly decreased. There is no significant difference between miR-205 and miR-205 (both) (*P* > 0.05), KDM4A mRNA and protein expressions significantly increased, and N-cadherin and MMP-9 protein expressions significantly decreased (*P* < 0.05). The above results indicate that hsa_circ_000 1429 negatively regulates the KDM4A gene by adsorbing miR-205, thereby promoting the migration and invasion of breast cancer cells.  Figure 6 shows hsa_circ_000 1429 adsorbed miR-205 to regulate KDM4A expression and inhibit breast cancer metastasis.

## 4. The Experimental Results Discussion

Breast cancer is a malignant tumor that occurs in the mammary epithelium or ductal epithelium, and its incidence is relatively high. Improvement of diagnosis and treatment methods can significantly reduce the mortality rate of the disease. Elucidating the pathogenesis of breast cancer has a very critical role in the treatment of breast cancer. More and more studies have shown that abundant circRNAs in mammals are closely related to neurological diseases, cardiovascular diseases, orthopedic diseases, and various cancers. Unlike linear RNAs, circRNAs form a closed continuous loop structure without 5'-3' polar or polyadenylated ends. CircRNAs are widely expressed in human cells and play an important role in the regulation of gene expression at the posttranscriptional level. There is only one literature showing that hsa_circ_000 1429 can promote breast cancer proliferation, migration, and invasion. However, there is no research report on the regulatory mechanism of hsa_circ_000 1429 in breast cancer. In this study, we first detect the expression of hsa_circ_000 1429 in normal mammary epithelial cells and breast cancer cell lines by culturing mammary epithelial cells MCF-10A and human breast cancer cell lines BT474, SKBr-3, ZR-75-30, and MCF7. The results show that the expression of hsa_circ_000 1429 is upregulated in breast cancer cells. hsa_circ_000 1429 can promote breast cancer cell proliferation, migration, invasion, and cell apoptosis.

CircRNAs play a key regulatory role in cancer, and most studies have shown that circRNAs have tissue and developmental stage-specific expression and act as microRNA-sponge RNAs to sequester microRNAs, thereby affecting the stability of target mRNAs and dynamically regulating mRNA translation. The paper passed the Circular RNA Interactome screening and revealed a binding site between hsa_circ_000 1429 and miR-205. The regulatory role of miR-205 in cancer is not clear. Some studies have shown that miR-205 plays a tumor suppressor role in tumors, inhibiting cancer proliferation, migration, and invasion. However, other studies have shown that miR-205 plays a role in promoting cancer. The study also finds that hsa_circ_000 1429 could act as a sponge RNA to competitively bind to miR-205. miR-205 overexpression inhibited the proliferation, migration, and invasion of breast cancer cells and promoted apoptosis. Our study confirms that miR-205 silencing can block the promotion of hsa_circ_000 1429 on breast cancer cell proliferation, migration, and invasion. It suggests that miR-205 may act as a tumor suppressor in breast cancer.

In order to further explore the regulatory mechanism of miR-205 in breast cancer, the study screens the possible target genes downstream of miR-205 through the bioinformatics website. The study finds that there is a binding site between KDM4A and miR-205, and the dual-luciferase reporter assay also confirms the targeted regulatory relationship between miR-205 and KDM4A. On further study, as a member of the JmjC family, KDM4A is found to be highly expressed in many types of cancers.

It has been shown that KDM4A involved in important biological processes such as gene transcription, cell cycle regulation, cellular senescence, DNA damage repair, and chromatin remodeling. Our study also shows that KDM4A overexpression blocked the promotion of hsa_circ_000 1429 on breast cancer cell proliferation, migration, and invasion.

## 5. Conclusion

In summary, the study finds that hsa_circ_000 1429 is upregulated in breast cancer cells and could upregulate the expression of miR-205 target gene KDM4A by adsorbing miR-205, which will promote breast cancer cell proliferation, migration, and invasion and promote breast cancer cell proliferation, migration, and invasion. This study explores the regulatory mechanism of hsa_circ_000 1429 in breast cancer, further improves the pathogenesis of breast cancer, provides a new research direction for exploring the pathogenesis of breast cancer, and provides new theoretical guidance for clinical treatment. However, the study does not conduct animal experiments yet and cannot further confirm the regulatory mechanism of hsa_circ_000 1429 in vivo. More experiments are needed to explore whether it is suitable for clinical treatment.

## Figures and Tables

**Figure 1:** Expression of hsa_circ_000 1429, KDM4A, and miR-205 in breast cancer cells.

**Figure 2:** hsa_circ_000 1429 adsorbed miR-205 to regulate KDM4A. (a) The binding site of hsa_circ_000 1429 and miR-205. (b) The binding site of miR-205 and KDM4A. (c) The binding relationship between hsa_circ_000 1429 and miR-205 verified by dual-luciferase experiment. (d) Dual-luciferase enzyme experiments verified the binding relationship between miR-205 and KDM4A. (e) RNA pull down experiment to verify that hsa_circ_000 1429 binds to miR-205. (f) RIP experiment.

**Figure 3:** MTT assay for cell proliferation.

**Figure 4:** Transwell assay to detect cell migration and invasion ability.

**Figure 5:** Flow cytometry is used to detect cell apoptosis in each group.

**Figure 6:** hsa_circ_000 1429 adsorbed miR-205 to regulate KDM4A expression and inhibit breast cancer metastasis.

**Table 1:** Primer sequences.

Gene name	Gene sequence (5′-3′) primer
hsa_circ_000 1429	F : CTCTCGTGGACCTCAGCCTC; R : GTCCAGGGAGTGCATGGTG
miR-205	F : GGGGAGGGGGAA AGTTCTA; R : GTGCGTGTCGTG GAGTCG
KDM4A	F : CTCATCAACTGTGGCGTCTG; R : TTAGTTTGCCCTTCATTTCC
GAPDH	F : GCACCGTCAAGGCTGAGAAC; R : TGGTGAAGACGCCAGTGGA
U6	F : GCTTCGGCAGCACATATAC TAAAAT; R : CGCTTCACGAATTTGCGTGTCAT

## Data Availability

The data used to support the findings of this study are available from the corresponding author upon request.
